# An Intelligent Health Monitoring Model Based on Fuzzy Deep Neural Network

**DOI:** 10.1155/2022/4757620

**Published:** 2022-08-18

**Authors:** Tianye Xing, Yidan Wang, Yingxue Liu, Qi Wu, Rong Ma, Xiaoling Shang

**Affiliations:** ^1^College of Basic Medicine, Changchun University of Chinese Medicine, Changchun 130117, China; ^2^Department of Information Engineering, College of Humanities & Information Changchun University of Technology, Changchun 130122, China; ^3^Department of Civil Engineering, Monash University, Wellington Road, Clayton, Victoria 3800, Australia; ^4^Shangfan School of Culture and Arts Co., Ltd, Yangguangxincheng, Tiedong, Jilin Siping 136099, China; ^5^Baoding Surveying & Mapping Center for House, Baoding Diangu Technology Center, 3-B -403, Hebei, China

## Abstract

An intelligent health detection model is a new technology developed under an artificial intelligence environment, which is of great significance to the care of the elderly and other people who cannot take care of themselves. This paper comprehensively reviews the structural health monitoring method based on an intelligent algorithm, introduces the application model of neural networks in structural health monitoring in detail, and points out the shortcomings of using neural network technology alone. On the basis of previous work, the genetic algorithm and fuzzy theory were introduced as optimization tools, and a new neural network training algorithm was constructed by combining genetic algorithm, fuzzy theory, and neural network technology for structural health monitoring research. Aimed at the shortcoming of insufficient samples for training neural networks based on experimental data, this paper proposes to use the finite element method to construct a genetic fuzzy RBF neural network after corresponding processing of the first six-order bending modal frequencies of the structure, so as to realize the localization and detection of delamination damage of composite beams. *Injury Assessment*. The experimental results of this paper show that the finite element method proposed in this paper can effectively carry out damage localization and damage assessment; compared with the traditional algorithm, the localization accuracy of this algorithm is improved by 20%, and the damage assessment performance is improved by 10%.

## 1. Introduction

To define what is health monitoring, we must first determine what is an injury. Health is relative to injury. In 2018, Bisson et al. conducted research on psychological impairment [1]. Injury refers to the destruction of the human body's skin, muscles, bones, organs, and other tissue structures caused by various external trauma factors and the local and systemic reactions brought about by it. The concept they put forward at that time formed the basic concept of damage mechanics and developed into the current discipline of damage mechanics on this basis. Kachanov believes that the expansion of microdefects is the main cause of damage. He defines the continuous variable *A*/*A*0, where *A* is the actual bearing area and *A*0 is the plain area (initial area). In 2017, Foertsch et al. conducted a study on the harm caused by the injury of the body in mice [2].

Structural damage can be defined as a whole or some parts of it, such as structural changes or declines in stiffness, strength, boundary, and connection conditions, which will affect the future performance of the structure system.

At present, due to the outstanding characteristics of composite materials such as high strength, high hardness, and low weight, composite materials have attracted more and more attention in many engineering applications (aerospace, automobiles, ships, railways, etc.), but due to composite materials, some uncertain factors in the preparation process make it impossible to fully guarantee its performance. In order to ensure the qualified rate of composite products, it is necessary to monitor during the manufacturing process to implement control. Composite materials must be composed of two or more material components with different chemical and physical properties in the designed form, proportion, and distribution, and there is an obvious interface between each component.

The latest developments have led to the latest developments in structure evaluation/detection technology, including structural health monitoring. The concept of structural health monitoring (SHM) is derived from bionics. Through labor, human beings use their smart intelligence and dexterous hands to make tools, thus gaining greater freedom in nature. It uses embedded or surface-attached sensor systems as the nervous system and the actuator as a muscle-like tissue that can sense and predict structural defects and damage. Fundamentally speaking, monitoring is to use a certain signal to interrogate the structural system and analyze the signal response to determine whether the structure has undergone some form of change, especially to know whether the measured change can hinder the normal operation of the system. The basic contents of health monitoring include the establishment of health records, dynamic health monitoring, evaluation of intervention results, and special health management and disease management services.

According to the literature [3], structural health monitoring can be defined as the following: In terms of expansion, structural health monitoring means nondestructive monitoring of the physical and mechanical properties of the structure. In a narrow sense, structural health monitoring refers to the strategy and process of damage identification and characterization of engineering structures, and structural damage refers to changes in structural material parameters and their geometric characteristics. Real-time monitoring of the overall behavior of the structure, diagnosis of the location and extent of the damage to the structure, and the service status, reliability, durability, and bearing capacity of the structure carry out an intelligent assessment to trigger early warning signals for structures in emergencies or serious abnormalities in the use of structures and to provide basis and guidance for structural maintenance, maintenance, and management decision-making.

In supervised learning, the problem of the previous multilayer neural network is that it is easy to fall into local extreme points, so the deep neural network is selected to detect the damage. The automated system for continuous monitoring, inspection, and damage detection can automatically report the status of the structure through the local area network or remote center. It is different from the traditional nondestructive testing technology (nondestructive evaluation, referred to as NDE). Therefore, historical data is very important, and the accuracy of the recognition is completely dependent on the sensor and the interpretation algorithm [4]. It can be said that health monitoring may transform the field of engineering structure safety monitoring, disaster reduction, and prevention.

From the previous introduction, it can be seen that structural health monitoring technology is a multidomain and interdisciplinary comprehensive technology, which involves civil engineering, dynamics, testing technology, and many other research directions.

## 2. Literature Review

### 2.1. Application of Artificial Network in the Health Monitoring of Composite Material Structure

The BP network is simple in structure and easy to implement, so it was first used in structural damage monitoring. The BP neural network is a multilayer feedforward network trained by error back propagation (referred to as error back propagation). Its algorithm is called the BP algorithm. Its basic idea is the gradient descent method, which uses gradient search technology to make the network. The error mean square error between the actual output value and the expected output value is the smallest. During the test, many researchers later developed different network models to monitor the damage to engineering structures or components. Among them, it has excellent generalization ability [3, 5–13], so it has great application prospects in the field of structural health monitoring.

In 1992, Jenq and Lee [14] used the BP network for damage detection of building structures. They used the frequency response spectrum before and after structural damage to train the network, used the measured structural response as the experimental sample, and conducted a numerical simulation study of a three-layer shear frame. In 1993, Nakamura et al. [15] used the BP neural network to successfully identify the damage degree of the five-story building structure without accounting for the measurement error (that is, the vibration test result is considered deterministic). In 1993, Maseras-Gutierrez et al. [16] used the first two-order bending mode frequencies of the cantilever beam as the input of the multilayer perceptual neural network and used the ideal output to identify the damage of the cantilever beam. In 1994, Catelsni and Ford [17] studied based on the damage detection problem of the multi-degree-of-freedom particle spring system of the BP network using natural frequency as the input parameter. Natural frequency refers to the frequency at which a system tends to oscillate without external force or damping. The oscillation of an elastic body without external force is called natural oscillation, and its corresponding frequency is the natural frequency. The results show that the recognition effect is better when the experimental sample falls near the training sample domain, and it may fail when it exceeds this range. In 1994, Stephens et al. used multiple damage indicators (maximum displacement, stiffness degradation, and energy dissipation) of the structure as the response of the structure under the action of an earthquake and established a neural network model to evaluate the safety level of the structure damaged by the earthquake. In the year 1995, Barai et al. used finite elements to simulate a model of a steel truss bridge accompanied by a vehicle passing by at a constant speed. The finite element method is a numerical technique for solving approximate solutions to boundary value problems of partial differential equations. When solving, the entire problem area is decomposed, and each subarea becomes a simple part. This simple part is called a finite element. The method of combining vibration method and artificial neural network is used to diagnose the damage to the steel truss bridge. In 1995, Rhim and Lee used the BP network model to study the damage monitoring of composite cantilever beams, using the transfer function of the structure as an input parameter and performed a numerical simulation. In 1997, Hanagud et al. used the BP network to identify delamination and stiffness drop damage in composite materials. Delamination damage is simulated by embedding Teflon film in the composite material, and different lengths represent different delamination sizes. Use a small hammer with a sensor to hit one end of the composite material, and use a piezoelectric sensor to measure the movement of the composite material. For state response, use the frequency response function as the input of the neural network and the delamination information as the output of the network. In 1997, Jenq and Lee used a BP neural network with an adaptive learning rate to predict the location (holes) in a composite laminated beam made of glass fiber reinforced plastic. They used measured data to modify the number theory of finite element calculation and use the first four-order modal frequencies of the structure as the input of the network and the size and location of the damage as the output of the network.

In 1997, Yaojun and Baoqi introduced the network to health monitoring. The frequency band of the original signal was decomposed into a series of properties of different frequency bands through wavelet transform, feature extraction was performed, and the wavelet neural network was used for learning. After training, the results show that this wavelet neural network can intelligently classify damage types and can still effectively diagnose when there is interference in the input pattern, and the system has a certain degree of robustness. In 1998, Nakamura et al. used the relative displacement between the layers of the structure and the relative speed between the layers as the input of the network, and the restoring force between the layers was taken as the output in 1995. The state before and after the restoration of the seven-story steel structure damaged in the Hanshin Earthquake corresponds to the damaged and nondamaged states, respectively, which verifies the effectiveness of the method. In 1998, Maseras-Gutierrez et al. discussed the use of piezoelectric sensors and neural networks to detect impacted composite materials. In 2000, Catelsni et al. used the RBF neural network to realize the automatic diagnosis and classification of faults. First, the neural network was trained with the fault database, and then, the new input data was put into the trained network classifier for pattern matching, which is the category of the fault. In 2001, Zang et al. used principal component analysis technology to preprocess FRF data, using compressed FRF data as the input of the neural network and outputting the damage and health status of the corresponding structure to monitor the structure. Principal component analysis technology, also known as principal component analysis, is aimed at converting multiple indicators into a few comprehensive indicators by using the idea of dimension reduction. In 2001, Haywood et al. analyze the characteristics of the dynamic strain response signal and use a neural network to identify the impact position and amplitude on the composite plate. In 2002, Watkins et al. used fiber optic sensors, and the BP neural network is used to predict delamination damage in composite beam structures. They used a MATLAB model based on the typical beam theory to obtain 1066 sets of fronts with different delamination sizes and positions. The fifth-order modal frequency is used as the training sample of the neural network. Experimental results show that the neural network predicts the location and size of delamination very closely.

In 2003, Chen et al. proposed that transfer function of the composite material structure is sampled to obtain training samples of the multilayer perceptron network, and the corresponding output is compared with the transfer function of the system, and the structural cracks and connection relaxation damage are studied. In 2003, Roopesh et al. used the vibration characteristic signal combined with the RBF neural network to study the damage to the helicopter rotor structure. In the same year, Yang et al. used to reduce the stiffness to a certain percentage to simulate the damage and combined with the RBF neural network to study the damage to free structures. In 2004, Dakai and others applied wavelet transform technology to the noise reduction processing of the input signal by the neural network and used the noise-containing output signal of the sensor fiber obtained in advance. After the network training is completed, the output signal of the sensing fiber to be detected is collected by the computer (through wavelet transform technology).

In 2004, Dakai and others applied wavelet transform technology to the noise reduction processing of the input signal and used the noise-containing output signal of the sensor fiber obtained in advance. After the network training is completed, the output signal of the sensor fiber to be detected collected by the computer (processed by wavelet transform technology) is input into the BP neural network to achieve simulation research on damage detection of the smart composite structure. In 2004, Shenchang et al. used drilling through holes to simulate the damage to a composite material laminated beam structure and used the RBF network that comes with the MATLAB toolbox to study the damage to the laminated beam structure.

They have fully improved the application of the BP network, and the BP network has been greatly developed in both the efficiency of the algorithm and the breadth of its application. However, they have not done much research on the application of the BP network in health detection and have not improved it much.

### 2.2. Application of Genetic Algorithm in the Health Monitoring of Composite Material Structure

The genetic algorithm introduces the principle of “natural selection” into the optimization process, because it is fundamental to optimization problems. There are no restrictions on it. The genetic algorithm is a search algorithm based on natural selection and population genetic mechanism, which simulates the phenomena of reproduction, hybridization, and mutation in natural selection and natural genetic process. The objective function and constraints are neither continuous nor differentiable, only that the problem can be calculated, and the search space is all over the solution space. Implied in it is a parallel computer system, so it is easy to get the global optimal solution, which can better overcome the difficulty of getting into the local minimum in the optimization process. Therefore, the genetic algorithm has strong vitality in the field of structural health monitoring. In 1996, Carlin et al. used the objective function of measuring frequency error and mode shape error as the fitness criterion to discuss and understand the influence of factors such as group size, crossover frequency, mutation frequency, and intersection point of the genetic algorithm on damage identification. For the numerical model for damage identification, in 1997, Ruotolo and Surace formulated the inverse problem of using the measured modal parameters to detect the position and depth of the cracks on the beam and then used genetic algorithms to solve this optimization problem. The genetic algorithm is said to be the most basic optimization algorithm. The principle is to compile the parent data and perform “inheritance and mutation” on it through a series of operations and continuously eliminate the individual data with low fitness to produce the global optimal solution. In 1998, Friswell et al. proposed a damage location method combining genetic algorithm with feature sensitivity. The method firstly analyzes the characteristic sensitivity of the structure, establishes an optimization objective function considering the natural frequency error, modal error, etc., uses the genetic algorithm to globally optimize the objective function containing the damage location information, and finally uses the simulated beam and the measured beam, respectively. The board verifies the method. In 2000, the genetic algorithm is used for global optimization to minimize the error between the characteristic frequency of the network output and the measured frequency. In 2000, Krawczuk et al. applied genetic algorithms to identify and locate structural damage in composite laminated beams. In 2001, Weijian et al. used genetic algorithms to process the dynamic information obtained from the experiment and proposed new improvement measures such as multiparent variable hybridization and variable fine-tuning, which were applied to multiple structures such as fixed-end beams, continuous beams, and frames. The damage recognition has achieved good results. In 2002, Koh et al. used a genetic algorithm with local search to analyze the measured excitation and response and identify structural parameters for damage identification. Numerical simulations of the slab/shell and aircraft wings show that the load position has a great influence on the recognition results. This method adaptively adjusts the deviation of the local search size through the global and local stages and has strong antinoise performance. In 2004, Xiangsen et al. used the change ratio of the first five-order modal frequency of the structure with the GA algorithm to train the network and studied the damage location of the structure.

## 3. Preliminaries

### 3.1. The Composition of the Health Monitoring System

The health monitoring system should include the following parts [5]:

1. Sensing System. Used to convert the physical quantity to be measured into an electrical signal.
2. Generally installed in the structure, the data of the sensor system is collected according to data and carried out preliminary processing.
3. Communication System. The collected data is transmitted to the center.
4. Center and Alarm Equipment. If an abnormality is found, an alarm will be issued. The system workflow is shown in Figure 1.

As shown in Figure 1, the five parts of the health detection system should be linked by the database, with the application layer as the center and the alarm device and the communication device as the auxiliary device. The sensing system is the underlying sensing structure.

### 3.2. Application of Structural Health Monitoring

There are many technical methods for structural health monitoring (SHM) [6–8]. According to different technical methods, structural health monitoring systems can be applied to (1) online monitoring of material properties in the manufacturing process and (2) various application purposes such as damage monitoring and integrity assessment of materials during use. Because the structural health monitoring technology has an advanced testing system and a high degree of automation, it can realize real-time online health monitoring of the structure, has good safety and reliability guarantees, and can save a lot of maintenance costs. With the continuous deepening of research on structural health monitoring systems, practical applications of structural health monitoring systems in the following fields have gradually become possible [9]. The structural health monitoring system includes stand-alone centralized online monitoring, distributed online monitoring, remote distributed online monitoring, and wireless sensor network monitoring. Structural health monitoring is widely used in intensive care units of hospitals. Because structural health monitoring can provide uninterrupted detection services and real-time detection of abnormalities, it can well detect the state of critically ill patients.

### 3.3. Optimization Problem

Many scientific and engineering problems can be reduced to optimization with constraint (optimization) questions; the general form of the mathematical model is [10]

(1) $$\begin{array}{c} \max{\left(\min\right)}_{z}=f\left(x_{1},x_{2},\cdots ,x_{n}\right). \end{array}$$

The constraints are *g*_*k*_(*x*_1_, *x*_2_, ⋯, *x*_*n*_){≤, = , ≥}0, *k* = 1, 2, ⋯, *m*, *z* is also called the objective function.

Optimization problems can be simply divided into linear optimization problems that are easy to solve and those that are more difficult to solve. For the nonlinear optimization problem, linear problems can be solved with very simple algorithms, and the optimal solution can be obtained in a limited number of steps. However, many of the problems encountered in engineering and other fields belong to the category of “difficult to solve” and cannot be solved using deterministic algorithms. Optimization has always been a hotspot in the mathematics community due to its inherent difficulties. For problem optimization, in the health detection system, you can define the optimal scheme of physical indicators and take the optimal scheme as the standard. It can be recognized as healthy within a certain range, and the alarm will be triggered if it exceeds the range.

### 3.4. Intelligent Algorithm

It is inspired by the laws of nature (biological world) and based on its principles, imitating algorithms for solving problems. Our common intelligent algorithms include simulated annealing, genetic algorithm, tabu search, neural network, beetle search algorithm, and sparrow search algorithm. With inspiration from nature, imitating its structure to invent and create, this is bionics. Intelligent optimization algorithms usually solve optimization problems. This algorithm makes it possible to search for the best solution within an acceptable computational cost. These algorithms or theories have some common characteristics, such as simulating natural processes. They are very useful in solving some complicated engineering problems.

The optimization algorithm is mainly composed of search direction and search step length. The selection of search direction and search step size determines the search breadth and search depth of the optimization algorithm. The search direction and search step length of the classic algorithm are determined by the local information (such as the derivative), so it can only perform an effective deep search for the part but cannot perform an effective breadth search, so it is difficult for the classic optimization algorithm to jump out of the local optimum. The intelligent optimization algorithm, in order to avoid falling into the local optimum like the classic optimization algorithm, uses a relatively effective breadth search, but doing so makes the amount of calculation unbearable when the problem is large. However, with the development of computer technology, a relatively large amount of calculation of intelligent algorithms has been solved, and great achievements have been made.

Classical optimization algorithms and intelligent optimization algorithms are iterative algorithms, but they are quite different [11], mainly as follows:

1. The classic algorithm uses a feasible solution as the initial value of the iteration, while the intelligent algorithm uses a set of feasible solutions as the initial value
2. The search strategy of classic algorithms is deterministic, while the search strategy of intelligent algorithms is structured and randomized
3. Most classic algorithms require derivative information, while intelligent algorithms only use information about the value of the objective function
4. Classical algorithms have strict requirements on the properties of functions, while intelligent algorithms do not have much requirements on the properties of functions
5. The calculation amount of the classic algorithm is much smaller than that of the intelligent algorithm. For example, for a large-scale optimization problem with poor function properties, the classic algorithm does not work well, but the general heuristic algorithm requires a large amount of calculation

All kinds of intelligent algorithms have unique advantages in solving optimization problems, and they all have common characteristics: they all simulate natural processes and solve problems. For example, a genetic algorithm draws on the evolutionary thought of survival of the fittest in nature, and a neural network directly simulates the human brain. They all have the following basic elements:

(1) Neighborhood, generating new feasible solutions

(2) The criteria for selecting and accepting solutions

(3) Termination criteria. Among them (4) reflects the ability of intelligent algorithms to overcome local optima

(6) Research on the convergence speed of intelligent algorithms, etc.

These technologies have decades of history, but at that time, these methods were not paid enough attention. It was because these methods were not very mature at that time, and the other was the limitation of computer software and hardware at that time, and these methods generally required a large amount of calculation and were difficult to obtain practical applications. With the development and popularization of computer technology, they have been developed by leaps and bounds in the last ten years. They have attracted the attention of experts and scholars in many fields and become an interdisciplinary research hotspot. In recent years, these methods have shown a trend of mutual integration, and their mutual complementation can enhance each other's abilities, so as to obtain more powerful expressions and the ability to solve practical problems. For example, researches on fuzzy neural networks, fuzzy classifier systems, and evolutionary design methods using genetic algorithms to optimize neural networks [12] all reflect the advantages of this fusion.

Intelligent computing will explore new concepts, new theories, new methods, and new technologies of intelligence, and all these will make major achievements in future development.

### 3.5. Artificial Neural Networks

The artificial neural network (ANN) is a high-tech research field, which is a hotspot of information science, brain science, neuropsychology, and other multidisciplinary intersections. It is based on the understanding of the human brain organization structure and operating mechanism. An engineering system simulates its structure and intelligent behavior. In the recent ten years, the research work on the artificial neural network has been deepened continuously, and great progress has been made. It has successfully solved many practical problems which are difficult to be solved by modern computers in the fields of pattern recognition, intelligent robots, automatic control, prediction and estimation, biology, medicine, economy, etc. and has shown good intelligent characteristics.

As shown in Figure 2, among them, *x*_*i*_ is the input signal that needs to be transmitted, *θ*_*i*_ thresholds, *W*_*ij*_ weighs, 4 is the external signal, that is, the bias signal, *s*_*i*_ is the output signal of the neuron node, *y*_*i*_ is the function of the neuron, and *f* is also often called the transfer function. The expression of the neuron model is

(2) $$\begin{array}{c} y_{i}=f\left(\underset{j}{\sum }W_{ij}x_{j}+s_{i}-\theta_{i}\right). \end{array}$$

## 4. An Intelligent Health Monitoring Model Based on Fuzzy Deep Neural Network

In the field of biology, the structure of the chromosome is a series of genes arranged hierarchically, some genes control other genes, some genes may be activated, and some genes may be dormant. Chromosomes can be expressed as a hierarchical structure including control genes and parameter genes. The parameter genes are at the lowest level, the control genes are at the upper level, and the lower-level gene string is controlled by the upper-level genes. The hierarchical genetic algorithm chromosome consists of two parts: (1) control gene and (2) parameter gene as shown in Figure 3.

The effect of the hierarchical genetic algorithm is different from that of the traditional genetic algorithm. Its operation can not only change the gene structure of this level but also cause a change in the gene structure of the next level. Therefore, the network parameters and topological structure can be optimized at the same time during the training process. Based on the characteristics of the hierarchical genetic algorithm, the patient's health indicators are optimized, and the indicators are modeled, with real-time changing data as input and the patient's health status as output.

### 4.1. Hybrid Hierarchical Genetic Algorithm to Optimize Neural Network

The neural network algorithm based on the hierarchical genetic algorithm can determine the neural network based on the sample data structure and parameters, but the convergence speed of the algorithm is slow in the learning process. Analyze what is used in this article. The structure of the RBF network and the WNN network shows that the output layer of the neural network is all linear neurons, which can be designed by the least square method. From the point of view of the genetic algorithm, this principle must be followed when encoding: the information in the encoding should not exceed the information necessary to express a feasible solution. The output weight of the network can be calculated by the least square method. Therefore, in the hybrid hierarchical genetic algorithm, only the parameters related to the hidden layer neurons are retained in the hierarchical chromosomes, as shown in Figure 4. The design of the output layer is completed in the evaluation function of the genetic algorithm.

### 4.2. Hybrid Hierarchical Genetic Algorithm Design

#### 4.2.1. Chromosome Coding Design

The coding design of chromosomes is divided into control gene and parameter gene design. The control gene adopts classic binary coding. Initialization is to set a maximum hidden layer node number *M* in advance; then, the coding of the control gene is a 0, 1 binary word of length *M*. string. The translation factor bi of the WNN is coded separately from the scale factor *a*. In order to facilitate the following comparison, the center width in RBFNN and the scale primer in WNN are initialized to real numbers in the interval [0, 1].

#### 4.2.2. Fitness Calculation

RBFNN is called the radial basis function neural network. It is a feedforward neural network with a single hidden layer and based on function approximation, which was put forward in the late 1980s. The training purpose of RBFNN and WNN is to make them have the simplest network structure while meeting certain accuracy requirements:

(3) $$\begin{array}{c} f=\frac{2N}{\left(a+{be}^{m/d_{n}}\right)\sum_{t=1}^{N}{\left(d_{i}-y_{i}\right)}^{2}}, \end{array}$$

where *N* is the number of samples. It can be seen that the smaller *m*, the larger *f* will be. According to experience, in the following example of delamination damage identification, the three undetermined coefficients of the fitness function are taken as *a* = 0.95, *b* = 0.05, *d* = 3, respectively.

*(1) Selection and Copy*. According to the different fitness of chromosomes in the population, reproductive opportunities are allocated. The probability that the individual with a large fitness value is selected is also higher. This article uses the roulette method (see 2.2.1.4 for specific calculations), which is also a typical selection operator.

*(2) Cross*. For this article, the chromosome is composed of two parts: gene and parameter gene, and the coding method is not the same, so this article proposes to use different cross operations for different parts.

*(3) Mutations*. Similar to the crossover operation, different mutation operations are used for control genes and parameter genes. For control genes, mutation operations are inversely calculated according to formula (2.7).

*(4) Adaptive Strategy*. The traditional setting method is static. This paper proposes to adopt the literature dynamic parameter setting method: *P*_*c*_ and *P*_*m*_ change with the change of fitness. When the fitness of each individual in the population tends to be consistent or locally optimal, *P*_*c*_ and *P*_*m*_ increase, and when the population fitness is relatively dispersed, *P*_*c*_ and *P*_*m*_ decrease; the expression is as follows:

(4) $$\begin{array}{c} P_{c}=\left\{\begin{array}{cc} \frac{P_{c1}-\left(P_{c1}-P_{c2}\right)\left(f^{\prime }-f_{\text{avg}}\right)}{f_{\max}-f_{\text{avg}}}, & f^{\prime }\geq f_{\text{avg}},\\ P_{c1}, & f^{\prime }<f_{\text{avg}}, \end{array}\right. \end{array}$$

(5) $$\begin{array}{c} P_{m}=\left\{\begin{array}{cc} \frac{P_{m1}-\left(P_{m1}-P_{m2}\right)\left(f_{\max}-f\right)}{f_{\max}-f_{\text{avg}}}, & f\geq f_{\text{avg}},\\ P_{m1}, & f<f_{\text{avg}}. \end{array}\right. \end{array}$$

*f* is the fitness value of the individual that needs to be mutated, and *f*_avg_ is the average fitness value of the current population.

## 5. Conclusion

This article first briefly introduces the concept, composition, and application prospects of structural health monitoring, then introduces intelligent algorithms, and focuses on the application of intelligent algorithms in structural health monitoring. Subsequently, the three intelligent algorithms mentioned in this article, namely, genetic algorithm, fuzzy clustering, and neural network technology, were used to conduct in-depth research on composite material structure health monitoring. The idea of combining these intelligent algorithms was put forward, making full use of the various algorithms and the advantages of each. Finally, the hybrid intelligent algorithm and computational mechanics are combined to monitor the delamination damage of composite materials. The main work completed in this paper and the conclusions obtained are as follows:

1. Send the experimental results of the modal analysis to the trained neural network for the identification of delamination damage. The identification results are given, and the results of several different methods are compared to verify the structure of the genetic fuzzy RBF neural network. There are broad application prospects in health monitoring research
2. This paper combines the successful combination of genetic algorithm, fuzzy theory, and neural network for theoretical research. And engineering application provides a new method, which has extremely important theoretical and practical significance
3. Use LMS' CADA-X modal analysis software to perform 10 modal analyses on each of the three composite test pieces that have been prepared, and take the average of the 10 analysis results as the test data of each test piece to verify. The effect of delamination on the modal frequency of the structure is discussed
4. Using the FEM method to calculate and simulate the first six orders of the test piece under different delamination damage conditions, bend the modal frequency, and use the experimental data to correct the calculated data to obtain the sample data and test data required for the network structure training in this paper

## Figures and Tables

**Figure 1:** Workflow of the health monitoring system.

**Figure 2:** Neuron structure model.

**Figure 3:** Chromosome structure of hierarchical genetic algorithm.

**Figure 4:** The parameters related to the hidden layer neurons are retained in the hierarchical chromosomes.

## Data Availability

No data were used to support this study.
